# Effects of Ultrasound-Guided Stellate Ganglion Block on Postoperative Quality of Recovery in Patients Undergoing Breast Cancer Surgery: A Randomized Controlled Clinical Trial

**DOI:** 10.1155/2022/7628183

**Published:** 2022-08-22

**Authors:** Xiuli Yang, Qixing Wu, Huan Wang, Yuwen Zhang, Xiaohui Peng, Lijian Chen

**Affiliations:** ^1^Department of Anesthesiology, The First Affiliated Hospital of Anhui Medical University, Hefei, Anhui, China; ^2^Department of Anesthesiology, Anhui Provincial Hospital, Hefei, Anhui, China

## Abstract

Surgery has been the primary treatment for breast cancer. However, instant postoperative complications, such as sleep disorder and pain, dramatically impair early postoperative quality of recovery, resulting in more extended hospital stays and higher costs. Recent clinical trials indicated that stellate ganglion block (SGB) could prolong sleep time and improve sleep quality in breast cancer survivors. Moreover, during the perioperative period, SGB enhanced the recovery of gastrointestinal functions in patients with laparoscopic colorectal cancer surgery and thoracolumbar spinal surgery. Furthermore, perioperative SGB decreased intraoperative requirements for anesthetics and analgesics in patients with complex regional pain syndrome. However, information is scarce regarding the effects of SGB on postoperative quality recovery in patients with breast cancer surgery. Therefore, we investigated the effects of SGB on the postoperative quality of recovery of patients undergoing breast cancer surgery. Sixty patients who underwent an elective unilateral modified radical mastectomy were randomized into two 30-patient groups that received either an ultrasound-guided right-sided SGB with 6 ml 0.25% ropivacaine (SGB group) or no block (control group). The primary outcome was the quality of postoperative recovery 24 hours after surgery, assessed with a Chinese version of the 40-item Quality of Recovery (QoR-40) questionnaire. Secondary outcomes were intraoperative requirements of propofol and opioids, rest pain at two, four, eight, and 24 hours after surgery, patient satisfaction score, and the incidence of postoperative abdominal distension. At 24 hours after surgery, global QoR-40 scores were higher in the SGB group than in the control group. Besides, in the SGB group, patients needed less propofol, had a lower incidence of postoperative abdominal bloating, and had higher satisfaction scores. Ultrasound-guided SGB could improve the quality of postoperative recovery in patients undergoing breast cancer surgery by less intraoperatively need for propofol and better postoperative recovery of sleep and gastrointestinal function.

## 1. Introduction

Rapid development of machine learning, practically deep learning, improves the accuracy of breast cancer detection [1], making it possible for breast cancer patients to receive early and effective treatments. Surgery has been the primary treatment for breast cancer [2], and modified radical mastectomy is acknowledged as a standard surgical treatment. However, early postoperative complications, such as pain [3, 4], general discomfort, fatigue, and sleep disturbances [5], significantly impede postoperative recovery, leading to extended hospital stays and high costs. Several clinical trials focused on breast cancer survivors, indicating drug administration, such as melatonin [6] and paroxetine [7], and stellate ganglion block (SGB) [7, 8] alleviated sleep disturbances and improved sleep quality. However, daily drug administration usually lasts several weeks or months, making it difficult for breast cancer patients to follow the prescription strictly. Furthermore, the effects of SGB were generally investigated during the rehabilitation period rather than during the perioperative period.

“Blind,” traditional SGB solely relies on anatomical landmarks, resulting in a high incidence of serious complications, including the unsatisfied level of block and direct puncture damage to the nerve structures. However, ultrasound-guided SGB is easy and safe to perform, improving the block quality and avoiding severe complications due to direct visualization of the needle position and the distribution of local anesthetics [9, 10]. SGB, a well-established anesthesia technique, is commonly used to treat sympathetically related pain in the upper limbs, head, and neck. Besides, ultrasound-guided SGB preceding general anesthesia enhanced the recovery of gastrointestinal functions in patients with laparoscopic colorectal cancer surgery [11] and thoracolumbar spinal surgery [12]. Furthermore, SGB could also relieve postoperative pain and decrease intraoperative requirements for anesthetics and analgesics in patients with complex regional pain syndrome [13].

However, little is known about the effects of ultrasound-guided SGB on the postoperative quality of recovery of patients with breast cancer surgery. Therefore, we planned to investigate the effects of ultrasound-guided SGB on the postoperative quality of recovery in patients undergoing breast cancer surgery. We hypothesized that patients who received an ultrasound-guided SGB before general anesthesia would have better postoperative recovery quality than those who did not.

## 2. Methods and Materials

This prospective, single-center, randomized controlled trial was conducted at the First Affiliated Hospital of Anhui Medical University in China. This study was approved by the Ethics Committee of the First Affiliated Hospital of Anhui Medical University (protocol number: PJ2020-05-09) and registered with the Chinese Clinical Trial Registry (Register number: chiCTR2000032658) on 5th May 2020, following the Helsinki Declaration and its revisions. Patients provided written informed consent before inclusion.

### 2.1. Patient Selection

Women with breast cancer who were scheduled for elective, unilateral, modified radical mastectomy were screened and recruited during preoperative assessment. The inclusion criteria were the following factors: aged 18–70 years and class I or II ranking based on the physical status evaluation system of the American Society of Anesthesiologists. The exclusion criteria were the following features: BMI greater than 30 kg m^−2^, a history of allergy to local anesthetics, infection near the puncture site, patients unable to communicate, and patients with chronic use of opioids.

### 2.2. Randomization and Masking

A list of randomized sequences was generated by an online random generator and sealed in opaque envelopes by staff not involved in the research. All participants were assigned randomly in a 1 : 1 ratio of a control group (ultrasound scanning only) and a group of patients who received ultrasound-guided SGB with 6 ml 0.25% ropivacaine (Astra Zeneca AB, Sodertalje, Sweden) (Figure 1). All patients, anesthetists, and outcome assessors were blinded to the study group allocation.

### 2.3. Intervention

Ultrasound-guided SGB was administered before general anesthesia in the preoperative area. Specifically, a right-sided single injection SGB was performed with real-time ultrasound (SonoSite Inc, Bothell, Washington, USA) by an attending anesthesiologist familiar with the ultrasound-guided nerve block. First, the patient was placed in the supine position with slight neck extension under appropriate monitoring. A 5–12 MHz linear transducer (SonoSite Inc, Bothell, Washington, USA) was placed at the sixth cervical vertebra (C6) level. After determining the location of the longus colli muscle, a 22 Gauge needle (KDL Medical Company, Zhejiang, China) tip was advanced posterior to the carotid artery, anterior to the longus colli muscle. Then, 6 ml of 0.25% ropivacaine was injected with the in-plane technique (Figure 1). Ten minutes later, patients were transferred to the operating room to induce general anesthesia. The presence of Horner's syndrome, including the decreased pupil size and ptosis (drooping of the upper eyelid), indicated the effectiveness of SGB.

### 2.4. Anesthesia Procedure

Standard monitoring and intravenous access were available. Standard monitoring included noninvasive blood pressure measurement, electrocardiography, peripheral pulse oximetry, partial pressure of carbon dioxide at the end of exhalation, temperature measurement, and bispectral index. Before anesthesia, all patients were given 10 mg dexamethasone for nausea prophylaxis. Total intravenous general anesthesia was sequentially induced with 0.1 mg kg^−1^ midazolam, 2.0 mg kg^−1^ propofol, and 0.5 *μ*g kg^−1^ sufentanil. Once the bispectral index value was less than 60, 0.2 mg kg^−1^ cisatracurium was intravenously administered to facilitate the insertion of a laryngeal airway mask (LMA). During the surgery, anesthesia was maintained with intravenous propofol infusion to maintain the bispectral index value between 40 and 50. Moreover, remifentanil was administered to keep the heart rate and blood pressure within 20% of the baseline. Additional sufentanil (0.2 *μ*g kg^−1^) and cisatracurium (0.05 mg kg^−1^) were intravenously administered as needed. After removing LMA, all patients were transported to the postanesthesia care unit (PACU) and then transferred to general wards if the postoperative steward score reached 6.

### 2.5. Outcome Measurements

The primary outcome was the global score of the quality of recovery, assessed with the Chinese version of the QoR-40 questionnaire. The questionnaire contains 40 questions that evaluate recovery in five aspects: nine items for emotional status, twelve items for physical comfort, seven items for psychological support, five items for physical independence, and seven items for pain. The total score is from 40, representing the poor quality of recovery, to 200, indicating excellent recovery. Each item is rated on a five-point scale: one (none of the time), two (some of the time), three (usually), four (most of the time), and five (all the time).

The secondary outcomes included intraoperative doses of propofol and opioids during general anesthesia, postoperative gastrointestinal function, and patient satisfaction scores measured with a ten-point scale (one = highly dissatisfied, ten = highly satisfied).

Intraoperative propofol and opioid doses, anesthesia time, surgery time, and recovery time were recorded, respectively. One team member who was blind to grouping recorded the scores of the QoR-40 questionnaire before and 24 hours after surgery. The visual analog scale score (zero = no pain and ten = worst pain imaginable) was used to evaluate at-rest patient postoperative pain intensity at discharge from the postanesthesia care unit, two hours, four hours, eight hours, and 24 hours after surgery. Two dimensions, namely, the first time for flatus and the incidence of abdominal distension, were used to evaluate the postoperative recovery of gastrointestinal function.

### 2.6. Sample Size

Power analysis of the two-tailed testing was based on the primary endpoint of the global QoR-40 score. A 10-point difference in the QoR-40 score after surgery was considered a clinically relevant enhancement in the quality of recovery [14, 15]. In our preliminary study, the global QoR-40 score, mean ± standard deviation (SD), was 160.7 ± 14.5 at 24 hours after the operation. Considering a 10% dropout rate, we enrolled 60 patients. The participant number was calculated using PASS version 15 (NCSS Statistical Software, LLC, Kaysville, Utah, USA) with *α* = 0.05 and *β* = 0.2.

### 2.7. Statistical Analysis

SPSS 21.0 software (SPSS, Chicago, Illinois, USA) was used for statistical analysis. The Shapiro–Wilk test was used to test the normal distribution of data. Parametric variables were reported as mean ± SD and analyzed between the groups using the independent-samples *t*-test. Nonparametric variables were reported as median (interquartile range (IQR)), and the Mann–Whitney *U* test was used to compare the two groups. Proportions were analyzed using *χ*^2^ analysis or Fisher's exact test as appropriate. All statistical tests were two-sided, and significance was accepted at *P* < 0.05.

## 3. Results

From May 2020 to December 2020, we conducted a single-center clinical trial at the First Affiliated Hospital of Anhui Medical University to investigate the effects of SGB on postoperative recovery in female patients with breast cancer surgery. Initially, 77 patients were assessed for study eligibility. Ten patients failed the inclusion criteria, and seven patients declined to enroll. Finally, 60 patients were enrolled and completed the study, with 30 in the ultrasound-guided SGB group and 30 in the control group (Figure 2).

Two groups were compared regarding demographics and clinical characteristics (Table 1). Global scores and each item score of the QoR-40 questionnaire before and after surgery are depicted in Table 2. Global QoR-40 scores at 24 hours after surgery were significantly greater in the ultrasound-guided SGB group (170.0 (166.8–173.0)) compared with the control group (160.0 (153.7–164.0)). Among the five dimensions of the QoR-40 questionnaire, only the scores of emotional status and physical comfort were significantly higher in the ultrasound-guided SGB group than in the control group (40.0 (39.0–42.0) vs. 37.0 (35.0–39.0), 49.5 (49.0–52.0) vs. 44.5 (41.0–47.3), respectively).

Intraoperative propofol, opioid consumption, and recovery time are depicted in Table 3. In the ultrasound-guided SGB group, the intraoperative need for propofol was considerably lower (*P*=0.006), and the recovery time was shorter in the ultrasound-guided SGB group (*P* < 0.001) as compared with the control group. However, the two groups had no significant differences in sufentanil or remifentanil consumption. Postoperative pain intensity at rest also did not significantly differ between the two groups (Table 4). Furthermore, fewer patients experienced postoperative abdominal bloating (*P*=0.024), and patient satisfaction scores were higher in the ultrasound-guided SGB group compared with the control group (*P*=0.016) (Table 5).

## 4. Discussion

This study demonstrated that after receiving a single ultrasound-guided SGB with 6 ml of 0.25% ropivacaine, significant improvements were found in the quality of recovery of patients who had an elective, unilateral, modified radical mastectomy. Specifically, patients in the ultrasound-guided SGB group had higher global QoR-40 questionnaire scores, greater satisfaction levels, and faster recovery of gastrointestinal function up to 24 hours after surgery.

The QoR-40 questionnaire is considered a reliable, multidimensional assessment tool [16]. Myles et al. considered that no less than a ten-point difference strongly indicated a clinically related improvement or deterioration [17]. Later, a 6.3-point difference was considered to represent a clinically associated change in the quality of recovery [18]. In our study, the postoperative global QoR-40 score was higher than ten points in the ultrasound-guided SGB group compared with the control group, which indicated that preoperative ultrasound-guided SGB was beneficial to the postoperative recovery of patients who had breast cancer surgery.

We did not find any complications resulting from SGB, mainly because ultrasound provided the direct monitoring of the needle advancement and the spread of local anesthetics. Left-sided SGB is typically used to manage refractory ventricular arrhythmia [19, 20]. In contrast, right-sided SGB exhibits a more effective antioxidative effect, reducing the catecholamine concentration in blood [21]. Therefore, we performed right-sided SGB in this study.

In our study, we found that patients in the ultrasound-guided SGB group had high emotional status and physical comfort scores, similar to earlier clinical findings. In a randomized controlled clinical trial, Wu et al. reported that SGB improved postoperative sleep by prolonging sleep time and improving sleep efficiency in patients with thoracoscopic surgery [22]. Similarly, Lipov et al. reported that SGB led to lower postoperative Pittsburgh Sleep Quality Index scores [7] and decreased night awakenings [8]. The autonomic nervous system is closely associated with sleep regulation. During different sleep stages, a dynamic balance is maintained between the sympathetic nervous system and the vagal nervous system [23, 24]. Patients with breast cancer have a higher extension of the sympathetic nervous system with a greater risk of experiencing sleep disturbances before and after surgery [25]. Sleep disturbance can negatively impact postoperative recovery [26, 27]. Although possible mechanisms of sleep disturbance are multifactorial, including severe anxiety and depression, immune response disorder, and circadian rhythm disorder [28], preoperative SGB can alleviate sleep disturbances by reducing sympathetic nervous activity, which benefits the postoperative quality of recovery in patients with breast cancer surgery.

In our study, we also found that the intraoperative need for propofol was dramatically decreased, probably due to the sedative effect of SGB. In an experimental study, the rats with SGB showed declined electroencephalogram activities [29], generally known as the depth of anesthesia. Besides, in the clinical trial with healthy volunteers, participants with SGB indicated decreased Observer's Assessment of Alertness/Sedation scores and bispectral index values [30]. The reduced intraoperative need for propofol could partially explain why the recovery time was shorter in patients with SGB. However, our study did not find the analgesic effect of SGB, contradicting the traditional notion that SGB could reduce sympathetic nervous system-related pain. The main reason is that perioperative pain in our study was mainly caused by surgery rather than being involved with high intensity of the sympathetic nervous system.

The postoperative period is associated with the disturbance of gastrointestinal function, such as bowel irritation and abdominal bloating. These problems occur mainly due to the imbalance between the sympathetic nervous system and the vagal nerve system attributed to operation stress, immobilization, and perioperative administration of opioids and narcotics [12]. Gastrointestinal morbidity can cause delayed feeding, anxiety, and sleep disturbance, leading to impaired patient recovery, prolonged hospital stay, and higher healthcare costs [31]. Early return of gastrointestinal function facilitates postoperative recovery of patients under general anesthesia. SGB can inhibit the excitation of the sympathetic nervous system, thereby restoring the balance of the autonomic nervous system and rebuilding the homeostasis of the neuroendocrine-immune system [32]. Furthermore, Zhao et al. reported that SGB relieved symptoms of chronic ulcerative colitis [33]. In our study, we found that patients in the ultrasound-guided SGB group had a lower incidence of abdominal bloating, indicating that SGB promoted the postoperative recovery of gastrointestinal function. Postoperative sleep and gastrointestinal function are governed by the autonomic nervous system and influence each other. Both have effects on the postoperative quality of recovery. Since the SGB inhibited the sympathetic system, the intraoperative stress was reduced, and then sleep and gastrointestinal function improved in the early postoperative period, which partially explained why the patient in the SGB group had a better quality of postoperative recovery.

Our study had some limitations. First, we only investigated the effects of ultrasound-guided SGB on female patients who had breast cancer surgery. Gender bias may influence the results. In addition, we only studied unilateral modified radical mastectomy; therefore, our findings cannot be generalized to other types of breast cancer surgery, like simple mastectomy or breast reconstruction. To design and more fully evaluate the effectiveness of ultrasound-guided SGB, we recommend additional multicenter studies that include larger numbers of participants and men who have other types of breast cancer surgery.

## 5. Conclusion

Ultrasound-guided SGB is likely to be associated with improved postoperative quality of recovery in patients with breast cancer surgery by less intraoperatively need for propofol and better postoperative recovery of sleep and gastrointestinal function.

## Figures and Tables

**Figure 1:** Horizontal ultrasound imaging of the stellate ganglion block. SCM, sternocleidomastoid muscle; IJV, internal jungle vein; CA, carotid artery; Lco, longus colli muscle, C6TP, transverse processes of the sixth cervical vertebra.

**Figure 2:** CONSORT flow of clinical procedures for the study. SGB, stellate ganglion block.

**Table 1:** Patient demographic and operative characteristics.

Variables	Control group (*n* = 30)	SGB group (*n* = 30)	*P* value
Age (years)	50.3 ± 6.8	51.4 ± 6.5	0.501
Height (cm)	161.2 ± 3.5	160.5 ± 4.0	0.476
Weight (kg)	59.5 ± 8.2	59.4 ± 5.9	0.943
Site of surgery (left/right)	11/19	13/17	0.598
ASA I/II	13/17	12/18	0.793
Duration of anesthesia (min)	106.7 ± 12.7	103.2 ± 12.6	0.271
Duration of surgery (min)	85.4 ± 13.7	82.2 ± 13.6	0.370

The variables are presented as mean ± SD. SGB, stellate ganglion block; ASA, American Society of Anesthesiologists; SD, standard deviation.

**Table 2:** Quality of recovery 40-item scores before and 24 hours after breast cancer surgery.

Variables	Control group (*n* = 30)	SGB group (*n* = 30)	*P* value
Before the surgery			
Global QoR-40 scores	184.0 (174.0–189.3)	184.5 (175.0–191.2)	0.739

24 hours after surgery	160.0 (153.7–164.0)	170.0 (166.8–173.0)	<0.001

Global QoR-40 scores			
Emotional status	37.0 (35.0–39.0)	40.0 (39.0–42.0)	<0.001
Physical comfort	44.5 (41.0–47.3)	49.5 (49.0–52.0)	<0.001
Psychological support	31.0 (29.7–31.3)	32.0 (30.0–33.1)	0.268
Physical independence	18.0 (16.0–19.0)	19.0 (17.0–20.3)	0.105
Pain	29.0 (27.7–31.3)	29.0 (28.0–30.2)	0.857

The variables are presented as median (IQR). SGB, stellate ganglion block; QoR-40, 40-item quality of recovery questionnaire; IQR, interquartile range.

**Table 3:** Intraoperative propofol, opioid consumption, and recovery time.

Variables	Control group (*n* = 30)	SGB group (*n* = 30)	*P* value
Propofol consumption (mg)	592.6 ± 87.8	531.8 ± 77.1	0.006
Sufentanil consumption (*μ*g)	37.6 ± 4.2	38.1 ± 4.8	0.651
Remifentanil consumption (*μ*g)	705.0 ± 96.1	680.3 ± 79.6	0.283
Recovery time (min)	23.1 ± 5.1	18.4 ± 3.9	<0.001

The variables are presented as mean ± SD. SGB, stellate ganglion block; SD, standard deviation.

**Table 4:** Postoperative visual analog score at rest.

Time points	Control group (*n* = 30)	SGB group (*n* = 30)	*P* value
PACU discharge	2.0 (1.0–3.2)	2.0 (1.0–3.0)	0.885
2 hours postoperatively	2.0 (1.0–3.0)	2.0 (1.0–3.0)	0.867
4 hours postoperatively	1.0 (0–2.0)	2.0 (1.0–2.2)	0.152
8 hours postoperatively	1.0 (0.7–2.0)	1.0 (0–2.0)	0.542
24 hours postoperatively	1.5 (1.0–2.0)	1.0 (0–2.0)	0.346

The variables are presented as median (IQR). SGB, stellate ganglion block; IQR, interquartile range; PACU, postanesthesia care unit.

**Table 5:** Postoperative gastrointestinal function and patient satisfaction score at 24 hours after breast cancer surgery.

Variables	Control group (*n* = 30)	SGB group (*n* = 30)	*P* value
First-time flatus time (hour)	8.0 (6.7–9.0)	7.0 (6.0–9.0)	0.380
Postoperative abdominal bloating	13 (43.3%)	5 (16.7%)	0.024
Patient satisfaction score	7.0 (5.7–8.0)	8.0 (7.0–9.0)	0.016

The variables are presented as median (IQR) or proportions. SGB, stellate ganglion block; IQR, interquartile range.

## Data Availability

The datasets used and/or analyzed during the current study are available from the corresponding author upon request.
